The article "Prediction of the Development Trend of the “Internet +” Logistics Industry under the “Belt and Road” Strategy" was published in 2022. Journal: Comput Intell Neurosci.

# Prediction of the Development Trend of the “Internet +” Logistics Industry under the “Belt and Road” Strategy

**DOI:** 10.1155/2022/4630146

**Published:** 2022-05-28

**Authors:** Chunhui Wen, Jinhai Yang, Zhuowu Zhang, Qianqian Guo, Haitao Xu

**Affiliations:** ^1^Economic College, Hunan Agricultural University, Changsha 410128, China; ^2^College of Business, Hunan University of Technology, Zhuzhou 412007, China; ^3^Cardiff Business School, Cardiff University, Cardiff CF10 3EU, UK

## Abstract

In order to accurately predict the development trend of the “Internet +” logistics industry in the context of the new period and to understand the circulation of the Internet and logistics between countries and the development dynamics of the economy, this paper will take the “Belt and Road” initiative as the research background and elaborate the specific development mode of the “Internet +” logistics industry and the corresponding strategies. Meanwhile, the development trend is evaluated based on its development data using the method of combined forecasting. The results show that the combined prediction results fluctuate within the range of 1, indicating a high degree of prediction accuracy. This is important for predicting the trend of development forces and adjusting the strategic approach and development direction.

## 1. Introduction

Internet technology is increasingly integrating logistics resources, and the traditional logistics industry is being embraced and transformed by the concept of “Internet +,” and new industry changes are imminent. At this stage, the domestic logistics industry is facing the challenges of global economic integration and the age of information technology. At the same time, the logistics industry should also actively respond to the challenge of optimizing the industrial chain model, effectively saving costs in the logistics industry, and achieving an overall improvement in management efficiency with the support of modern science and technology [1–3].

The most obvious feature of this initiative is its great potential and long span, making it the largest international development initiative spanning a wide range of distances. In the early years of the Belt and Road concept, our close ties and cooperation with countries in South East Asia and beyond led to an increase in the volume and scale of export trade. At the same time, the volume of our imports also increased. Most of them have close cooperation with China, both in terms of transport construction and in sharing energy and information [4–6]. The expanding scope of cooperation also brings more opportunities for investment and development for countries along the route. As of 2015, China has already made cooperation and investment plans with more than 50 countries along the road. After a period of observation and analysis, it is not difficult to find that some of the countries along the Belt and Road are not well developed in terms of infrastructure, the most important roads, railways, and other basic modes of transport, which undoubtedly brings more opportunities for China compared to our complete transport infrastructure and system [7–12]. The “Internet +” action plan has been incorporated into the government work report for the first time in 2015, Keqiang Li declared. If so, many industries would benefit from the plan, and there is no doubt that it is a great chance for industrial upgrading and technological innovation. “Internet + agriculture” will allow traditional agricultural methods to evolve digitally, greatly increasing the efficiency of agricultural production, and the combination of agriculture with the Internet will attract more young people to invest in traditional agricultural production, injecting more vitality and modernity into the development of new agriculture. “Internet + retail” is an effective combination of physical shops and online shops. The rise of the term e-commerce has given a new market and vitality to traditional retail methods. The concept of “Internet +” is a broad one, so it is interesting to see how the integration of “Internet +” with the transport and logistics industry will lead to a collision of sparks. The term “resource sharing” has been around for a long time and is popular in the fast-paced life we live. Our space is getting smaller and smaller, and we have to share our limited resources to seek common progress. Railways, roads, and sea transport are all essential platform tools for logistics, and the sharing of resources and interconnectivity between regions is the essence of the logistics industry. The combination of the concept of “Internet + logistics” will also bring better prospects for the “Belt and Road” strategy.

The meaning of “Internet +” is a strategic approach to regional economic development by using the Internet as an important basis for development and organically combining it with traditional and real industries. China has a population of more than 1.4 billion, accounting for 35% of the international economy. To be in an advantageous position in international competition, it must have a strong logistics capacity. It is also important to note that “Internet +” is also the main direction of future information development. With the innovation and improvement of network technology, it has effectively changed the way people live and work, so people should attach great importance to this change and should correctly perceive the important role of the Internet concept. The logistics industry based on “Internet +” should not only have the necessary Internet concepts but should also use modern technology in a reasonable way in the actual development of the industry. At present, the domestic logistics industry has initially integrated with the Internet and formed a marketing model in the form of the Internet in the logistics industry. To a certain extent, this has expanded the scope of online sales. The future development of the “Internet +” logistics industry provides certain opportunities. This has laid a foundation for industrial upgrading and has further strengthened the international competitiveness of the domestic logistics industry.

## 2. Strategies for the Development of “Internet + Logistics” Industry under the “Belt and Road” Initiative

1. The way initiative is the best national economic development initiative, building a closed-loop structure for regional economic development. There are many emerging economies and developing countries along the road initiative, which has become a fast-growing region for trade and cross-border investment in the international arena at this stage [13–17]. The development of the “Internet +” logistics industry based on the “way” initiative must be approached from a macro perspective, and through the flexible use of macroeconomic policies, a logistics network with more modern characteristics must be formed. In this process, the logistics base and modern technology must be used scientifically and rationally to achieve the overall optimization of logistics resources allocation. As the Belt and Road initiative is relatively long, it is important to connect countries and industries to each other in order to further promote sustainable industrial and economic development. On this basis, infrastructure development should be further promoted and a more comprehensive infrastructure network should be built. For developing and emerging countries, intercountry logistics development is hampered by relatively poor infrastructure. In the context of implementing the “Belt and Road” initiative, cooperation between countries will continue to deepen and achieve comprehensive collaboration, focusing on the role of information infrastructure construction, effectively promoting the comprehensive development of broadband networks, saving the cost of Internet development, and providing Internet services for logistics enterprises in the process of development.
2. At this stage, the global economy is in a period of transformation and upgrading, and most regional economic layout is gradually deepening, so the importance of the trade and logistics industry in economic development is highlighted. In this context, the logistics industry should actively adopt an innovation-driven model in order to achieve further development. In this process, the logistics industry should develop its innovation capabilities and enhance the degree of integration with the Internet + in order to build an innovative development environment. Furthermore, the industry's development standards and norms should be strictly formulated, and the “Internet +” information technology should be treated as a prerequisite for development and effectively applied to the industry's development needs. Information resources in the logistics industry should be shared, and relevant logistics enterprises should be actively guided to optimize their layout in order to achieve further development of the logistics industry. Along with the development of new information technology, the domestic intelligent logistics industry has achieved comprehensive changes, and the implementation of the integration of the supply chain has gradually become the development goal of the logistics industry. According to the actual survey results, the emptying rate of trucks in domestic road transport exceeds 40%, while the interval between parking and distribution is about 72 hours, making the problem of waste of resources and environmental pollution more serious. After the use of Internet technology, the problems of truck matching can be solved. Taking a road port as the object of study, the distribution time of trucks has been shortened by about 5 hours, which makes the cost investment of manufacturing enterprises and trade enterprises in logistics reduced by nearly 40%. The development of the logistics industry is also inseparable from the organic integration of resources, and the integration of enterprise resources and industry association resources can provide a strong guarantee for the sustainable development of the industry. The entire logistics + Internet operation process is shown in Figure 1.

## 3. Construction of a Predictive Evaluation System Based on Existing Models

### 3.1. The Connotation of Internet + Logistics

In the context of regional economicization, the evaluation index system of regional “Internet + logistics” cross-border development is constructed based on the five development forces: cross-border information flow development force, cross-border commercial flow development force, cross-border logistics development force, cross-border capital flow development force, and cross-border service flow development force, which can provide environmental analysis methods and tool support for the research of enterprises' “Internet + logistics” cross-border connection strategies.

Internet + logistics cross-border connectivity is the process of cross-border business activities in which enterprises rely on the cross-border connectivity function of the Internet + and the services of cross-border trade-related industries to sell their products or services to overseas markets across national borders. The better the conditions, foundation, and environment for Internet + logistics cross-border connectivity between regions (countries), the higher the quality of cross-border trade-related services that can be provided. The more favorable it will be for enterprises between two regions (countries) to sell their products or services to each other's markets through Internet + logistics cross-border connections. According to the study, the stronger the cross-border connectivity and cross-border resource integration capabilities of enterprises in a region based on the same level of digital infrastructure such as cloud, network, and terminal, the stronger the level of Internet + development power of the region. Based on the value creation process of cross-border connection of enterprises' Internet + logistics, this paper defines the cross-border development power of regional Internet + logistics as “the degree of facilitation and liberalization of cross-border connectivity between enterprises in a region (country or location).” For enterprises, the more convenient and free the cross-border connection of enterprises between regions (countries or locations), the greater the cross-border development momentum of regional Internet + logistics, and the more favorable the development of cross-border connection of enterprises through “Internet + trade” to explore each other's markets. Conversely, the more costly and restrictive the cross-border connection of enterprises between regions (countries or locations), the weaker the cross-border development momentum of regional Internet + logistics, and the more unfavorable it is for enterprises to develop each other's markets through the cross-border connection of “Internet + trade.” The connotation of regional Internet + logistics development power is shown in Figure 2.

### 3.2. Comprehensive Evaluation System of Regional “Internet + Logistics” Cross-Border Development Power

1. Regional “Internet + logistics” cross-border development force is a complex and comprehensive concept. Therefore, indicators should be designed systematically and comprehensively. The selected indicators should have a strict internal logical relationship and integrate the indicators to form a systematic and comprehensive organic evaluation system [18, 19].
2. The indicators should be integrated to form a systematic and comprehensive organic evaluation system, so as to conduct a comprehensive and systematic evaluation of the cross-border development power of the regional “Internet + logistics.”
3. Principle of scientificity. The selection of evaluation indicators should be based on the practical experience of domestic and foreign development and the existing research results of scholars and combined with the theory of cross-border connection mechanism of enterprise “Internet + logistics” in this paper.
4. The principle of comparability and quantifiability. The evaluation system of regional “Internet + logistics” cross-border development capacity involves horizontal comparison and vertical comparison in time series of multiple countries and regions. Therefore, when setting the indicators, we should fully consider the consistency of the indicators in the scope of research, the uniformity of the measurement methods, statistical years and data sources of the same indicators, and the selected indicators should be quantifiable and comparable and not too abstract.
5. Principle of hierarchy. The concept of regional “Internet + logistics” cross-border development power involves multiple levels of content. In order to evaluate the level size of regional “Internet + logistics” cross-border development power more clearly and comprehensively, the evaluation system should be constructed with multiple perspectives and levels in mind, reflecting different evaluation systems and the variability of the scale and characteristics of different regional Internet + logistics cross-border development power [20, 21].
6. The principle of data availability and reliability. In the process of developing the indicator system, we should not only consider the rationality of the indicators but also their availability and reliability. The indicators selected in this paper all come from the public panel data authoritatively released by the World Bank, the World Monetary Fund, the China Bureau of Statistics, the China Customs, and other institutions, as well as authoritative databases such as Wind and CSMAR. The amount of data is sufficient. This paper measures the regional “Internet + logistics” from two dimensions: “Internet carrier (A_1_)” and “Technical support (A_2_).” The development power of cross-border information flow (A) is shown in Table 1. In the secondary evaluation indicators, “Internet carrier (A_1_)” reflects the degree of Internet technology application between regions, while “Technology support (A_2_)” reflects the Internet basic science and technology development capability between regions. For the three-level indicators, the indicators including “Internet penetration rate (A_a1_),” “Fixed broadband subscriptions (A_a2_),” “Mobile phone usage (A_a3_),” and “ Number of secure Internet servers (A_a4_)” are used to measure the secondary indicator “Internet carriers (A_1_)”; the indicators including “Exports of high-tech products (A_a5_),” “Technology readiness (A_a6_),” and “Innovation capacity (Aa_7_)” are selected to measure the secondary indicator “Technical support (A_2_).”

### 3.3. Measurement of Indicator Weights

In the field of economic management, the methods used to determine the weights of the indicator evaluation system are: (1) principal component analysis, in which variables that carry overlapping information in the study are deleted to create as few new variables as possible, and the new variables are not correlated with each other; (2) equal weight method, in which the total weight is set to 1, and the indicator system has a total of *n* indicators, and each indicator has a weight of 1/*m*; (3) Delphi analysis; (4) AHP hierarchical analysis, which is a combination of qualitative and quantitative analysis that allows for a logical approach, experience, insight, and intuition to analyze and evaluate problems with large uncertainties; and (5) the lower the information entropy of an indicator, the lower the uncertainty of the indicator. Therefore, its weight will be greater. Conversely, the same applies. Compared with the mainstream comprehensive evaluation research methods mentioned above, this paper argues that the dimensionality reduction method of principal component analysis puts too much emphasis on avoiding the covariance of data, reduces some indicators, and loses some information, which causes the whole index system could not reflect the overall economic management.

The equal-weight method gives equal weights to each indicator and ignores the important differences between indicators. The Delphi and AHP methods rely too much on the subjective decisions and judgments of the researcher. Therefore, the weights obtained are highly subjective and lack scientific persuasiveness. The quantitative data in this paper are all from authoritative official statistics, so they are truly comparable.

The entropy method has the following advantages in this study: (1) it is more objective and has better generalisability. The purpose of evaluating the cross-border development power of regional “Internet + logistics” is to better help Chinese enterprises develop differentiated cross-border connectivity strategies according to local conditions. Therefore, the weighting of each indicator in the evaluation system must be objective and the entropy method. (2) It matches the scope of application with the measurement method.

The regional “Internet + logistics” cross-border development force system measured in this paper involves multi-level, multi-dimensional, and multi-indicators. The study shows that the entropy value method is suitable for providing objective weights for the combined evaluation system. Therefore, the entropy value method is used to determine the weights of regional “Internet + logistics” cross-border development evaluation indicators.

The procedure is as follows: the first step is to standardize the data. The data are collected by year, and the collected index data have different meanings and units. In order to carry out a scientific comparison and analysis, the weights are calculated in this paper. In order to carry out a scientific comparative analysis, this paper unifies the units of measurement of the raw data of the data indicators and standardizes the obtained indicator data with Min-max. The min-max standardization formula for positive indicators and the min-max standardization formula for negative indicators are as follows:

(1) $$\begin{array}{c} x_{ij}^{\prime }=\frac{x_{ij}-\min\left\{x_{j}\right\}}{\max\left\{x_{j}\right\}-\min\left\{x_{j}\right\}}, \end{array}$$

(2) $$\begin{array}{c} x_{ij}^{\prime }=\frac{\max\left\{x_{ij}\right\}-x_{ij}}{\max\left\{x_{j}\right\}-\min\left\{x_{j}\right\}}, \end{array}$$

where *x*_*ij*_′ refers to the data after min-max standardization, *x*_*j*_ represents the original data of the *j*^th^ indicator of the *i*^th^ study object, max{*x*} represents the maximum value of the *j*^th^ indicator element data, and min{*x*} represents the minimum value of the *j*^th^ indicator element data, and min-max standardization method is a linear transformation of the original data. The standardization method is a linear transformation of the original data, in which a raw indicator of study object *i* is mapped to *x*′*y* in the interval [0,1] through standardization, and the processed data form an attribute decision matrix *M*, with *Am* representing the contribution of the *j*^th^ indicator in the indicator evaluation system in a given year.

(3) $$\begin{array}{c} M=\left\{\begin{array}{c} A1\\ A2\\ A3\\ \cdot \cdot \cdot \\ A4 \end{array}\right\}\left[\begin{array}{cccc} x_{11} & x_{12} & \cdots & x_{1m}\\ x_{21} & x_{22} & \cdots & x_{2m}\\ x_{31} & x_{32} & \cdots & x_{3m}\\ \cdots & \cdots & \cdots & \cdots \\ x_{m1} & x_{m2} & \cdots & x_{mm} \end{array}\right]\left(i=1,2,\ldots ,j=1,2,\ldots ,Am=\sum_{i=0}^{n}x_{ij}^{\prime }\right). \end{array}$$

In the second step, the weight of the dimensionless data is derived.

*P*_*i,j*_ denotes the share of *Am* in the year under indicator *j* for region *i*, calculated as follows:

(4) $$\begin{array}{c} P_{i}{\;}_{j}=\frac{x_{ij}^{\prime }}{\sum_{i=1}^{n}x_{ij}^{\prime }}\left(i=1,2\ldots ,n;j=1,2\ldots ,m\right),\\ P_{ij}=P_{nm}=\left[\begin{array}{c} P_{11\;}\;P_{12}\;P_{13}\;\cdots P_{1m}\\ P_{21}\;P_{22}\;P_{23}\;\cdots P_{2m}\\ \cdots \;\cdots \;\cdots \;\cdots \;\\ P_{n1}\;P_{n2}\;P_{n3}\;\cdots P_{nm} \end{array}\right]. \end{array}$$

In the third step, the entropy value and the information utility value of the *j*^th^ indicator are calculated. The formula for calculating the entropy value *E* of the *j*^th^ indicator is shown specifically in following equation:

(5) $$\begin{array}{c} E_{j}=-K\sum_{i=1}^{m}P_{ij}\ln\;P_{ij}\left(j=1,2\cdot \cdot \cdot ,m\right), \end{array}$$

where ln is the natural logarithm, *E* is greater than is equal to 0, the constant *K* = 1/ln (*n*), and *n* is the number of evaluation objects.

In the fourth step, the information utility value of the *j*^th^ indicator is calculated. The size of the indicator weight is directly influenced by the information utility value of the indicator; the larger the entropy value of the indicator, the smaller the information utility value.

The higher the entropy value of the indicator, the higher the information utility value. The greater the difference, the greater the information utility value, the greater the contribution of the indicator to the evaluation system, and vice versa. The information utility value of the *j*^th^ indicator is expressed as follows:

(6) $$\begin{array}{c} d_{j}=1-E_{j}. \end{array}$$

In the fifth step, the weight of the *j*^th^ indicator is calculated. The formula for calculating the weight *W* of the *j*^th^ indicator is as follows:

(7) $$\begin{array}{c} W_{j}=\frac{d_{j}}{\sum_{J=1}^{n}d_{j}}. \end{array}$$

In the sixth step, the composite evaluation value of the *j*^th^ indicator of the *i*^th^ study object is calculated. The sum of the product of the standardized data of each indicator and its weight is its composite evaluation value. The formula for calculating the composite evaluation value *S*_*ij*_ of the *j*^th^ indicator of the *i*^th^ research subject is as follows:

(8) $$\begin{array}{c} S_{ij}=W_{j}\times x_{ij}^{\prime }. \end{array}$$

In the first step, after determining the standardized data and corresponding weights, the indices of the five submodules of the regional “Internet + logistics” cross-border development index are measured by the multi-objective linear weighting method, including the cross-border information flow development index, cross-border commercial flow development index, cross-border logistics development index, cross-border capital flow development index, and cross-border service flow development index.

(9) $$\begin{array}{c} \text{Cross}-\text{border Information Flow Index}:\;A_{1}=\sum_{j=1}^{a}W_{j}x_{ij},\\ \text{Cross}-\text{border Commercial Flows Index}:\;B_{1}=\sum_{j=1}^{b}W_{j}x_{ij},\\ \text{Cross}-\text{border Logistics Index}:\;C_{1}=\sum_{j}^{c}W_{j}x_{ij},\\ \text{Cross}-\text{border Financial Flows Index}:\;D_{1}=\sum_{j=1}^{d}W_{j}x_{ij},\\ \text{Cross}-\text{border Services Index}:\;E_{1}=\sum_{j=1}^{e}W_{j}x_{ij}. \end{array}$$

The number of indicators at three levels in the cross-border credit flow development capacity module is *a*. The number of indicators at three levels in the cross-border commercial flow development capacity module is *b*. The number of indicators at three levels in the cross-border logistics development capacity module is *c*. The number of indicators for the three levels in the cross-border financial flow connectivity module is *d*, and the number of indicators for the three levels in the cross-border service flow development capacity module is *e*. The total number of indicators is *M* = *a* + *b* + *c* + *d* + *e*. The second step is to use the comprehensive index method to measure the total index of regional “Internet + logistics” development power, and the formula for calculating the total index of regional “Internet + logistics” cross-border development power of the *i*^th^ research object is as follows:

(10) $$\begin{array}{c} ECI=A_{i}+B_{i}+C_{i}+D_{i}+E_{i}=W_{j}x_{i}{\;}_{j}. \end{array}$$

The above calculation process enables a systematic evaluation of the development trend of “Internet + logistics,” and in the following sections, a detailed forecast of the development trend is given.

## 4. Analysis and Evaluation of Development Trends

There are 64 countries and regions along the Belt and Road in addition to China. According to the purpose of the study, especially considering the availability and completeness of the research data, the scope of the sample was determined as 64 countries along the road.

From the perspective of each country's development power, the situation varies from country to country, but the development trend and the development increment are basically the same pattern, as shown in Figures 3 and 4.

The growth rate of each region shown in Figures 3 and 4 and the fluctuation of the growth rate of each region over the years show that different countries and regions have different logistics levels and increments due to their own technology and Internet level. The Czech Republic and Thailand show high growth rates in terms of regional growth rates. At the same time, it can be seen that as the years go on, the overall growth rate also shows an upward trend, with 2019 being greater than 2018 and even greater than 2017. This is further illustrated by the year-on-year growth rates and growth intervals for different years, as well as the distribution of total volumes, as shown in Figures 5 and 6.

The development efficiency and speed of development as well as the total amount of development can be seen in Figures 5 and 6, which basically show an increasing trend. Preprocessing the sample data for prediction shows that all the data fluctuate at (0.05, 0.05) as the center. Its highest growth total is at 10 billion, in terms of the maximum growth rate at 0.1. In the process of optimising the distance between the training sample and the prediction node, the coincidence function *ci*(*j*) at the prediction node is first constructed by using the relative error *Ei*(*j*):

(11) $$\begin{array}{c} ci\left(j\right)=1-Ei\left(j\right), \end{array}$$

where *i* is the ordinal number of the single prediction model and *j* is the ordinal number of the prediction node. According to *ci*(*j*), the prediction effect at the corresponding prediction node can be evaluated. The larger the coincidence value is, the better the prediction effect is, relatively; on the contrary, the worse the prediction effect is, relatively. Secondly, as mentioned before, the closer the distance, the greater its contribution value or freshness to the prediction node; conversely, the smaller the contribution value or freshness. Therefore, the freshness function *f*(*t*) is introduced again, and its calculation formula is *f*(*t*) = 1/*t*2; in equation (12), *t* is the distance between the ample and the prediction value. According to (12), the greater the distance between the sample and the prediction value, the smaller the value of the freshness function *f*(*t*), which is consistent with its meaning. Finally, *ci*(*j*) and *f*(*t*) are then used as the basis to construct a comprehensive evaluation function *li*(*j*)*t* considering the distance between the samples and the prediction value.

The formula for its calculation is

(12) $$\begin{array}{c} li\left(j\right)t=F\left(j\right)ci\left(j\right)=\left(\frac{1}{t2}\right)*\left[1-Ei\left(j\right)\right], \end{array}$$

where *li*(*j*)*t* not only reflects the influence of the distance between the training sample and the prediction node on the prediction result but also effectively reflects the degree of fit at the corresponding prediction node, which has a strong comprehensiveness. At the same time, the larger *li*(*j*) is, the better the prediction effect is; on the contrary, the worse the prediction effect is. Firstly, as *li*(*j*)*t* is mainly used for the evaluation at the corresponding prediction node, which can then be used to solve for the local combination weights *wJ*(*i*); the solution formula is as follows:

(13) $$\begin{array}{c} wJ\left(i\right)=\frac{li\left(j\right)}{\sum li\left(j\right)}, \end{array}$$

where *n* is the number of single models and *N* is the length of the distance between the training samples and the prediction nodes. Secondly, considering that the local combination weights already contain the prediction accuracy evaluation and thus focusing on the stability of the prediction results in the process of constructing the global combination weights *wQ*(*i*), the solution formula is expressed as follows:

(14) $$\begin{array}{c} wQ\left(i\right)=\frac{qi}{\sum qi}, \end{array}$$

where *qi* is the inverse of the variance value of the corresponding single model prediction result. Finally, the aforementioned has been calculated to obtain *wJ*(*i*) and *wQ*(*i*), needfurther combination of the two types of weights to realize the optimization of the local combination idea and the global combination ideas, and combined with the relevant literature research results, it is concluded that the cumulative superposition idea has a relatively better combination effect, and then *wJ*(*i*) and *wQ*(*i*) should be multiplied to obtain the combination of prediction of the base evaluation index *m*(*i*) as *m*(*i*) = *wJ*(*i*)*wQ*(*i*); the larger the value of *m*(*i*), the better the prediction effect of the single model, which is then normalized, and the resulting normalized value *wG*(*i*) can be used as the final combination weight of the combination prediction model in this paper, and its solution formula is *wG*(*i*) = *m*(*i*)*∑ni* = *1m*(*i*). Through the above stepwise optimization, the shortcomings of the traditional combination forecasting method are effectively overcome.

The results of the data training are shown in Figure 7.

From the growth rate of different regions shown in Figure 7, the growth rate of each region in the development of “ Belt and Road” Internet + logistics is fluctuating trend around 0.05: some regions are higher than 0.05, and some are lower than 0.05. The change of the development power error distribution point can be seen that the training error range of the model is about 1, which indicates that the results of the model are more accurate. On this basis, the predicted development force for the following years basically shows a fluctuating trend, with a suspected peak in 2026 and then decreasing. This is shown in Figure 8:

Figure 8 shows the evolution of the TDP growth rate, reflecting the trend of the total growth rate. It is clear that there will actually be a slow decline during 2019–2023, which is directly related to the slowdown in logistics and other industries due to the occurrence of the epidemic. And there will be a peak situation in the period 2024–2026. Thereafter, there will be a rapid decline. The reasons for this decline need to be further tested. However, the model is still relatively accurate for the current situation. Figures 9 and 10 are based on our further description of country development and related data.

Figures 9 and 10 show the growth rates of different countries in the “Internet + logistics” model and the development of Belt and Road. Through Figures 9 and 10, we can see that the Internet logistics industry in Asia is growing well and accounts for a larger share of the Belt and Road environment, while other countries are also growing to some extent but have not yet gained significant momentum.

## 5. Conclusion

Through the evaluation of the development trend of “Internet +” logistics, it can be determined that the combined forecasting method in this paper has a high prediction accuracy. Compared with traditional forecasting models, it has more obvious superiority. Its prediction results show high accuracy and can predict the trend force of development. At the same time, this study also helps further deepen and promote the systematic and comprehensive construction of “Internet +.” The findings of this paper can be further applied and sublimated by exploring the following aspects.

Firstly, in building and forming a complete strategic management theory of cross-border docking of “Internet+” enterprises, it is necessary to explore and verify the cross-border docking mechanism of enterprise “Internet + trade.” At the same time, the research horizon is improved to form the theoretical system of enterprise “Internet+” cross-border docking.

Secondly, a comprehensive evaluation system of regional “Internet +” cross-border connections should be established. On the one hand, the comprehensive evaluation index system of regional “Internet + trade” cross-border connection should be further improved. Besides, a comprehensive evaluation system of regional “Internet+” cross-border connection with a broader research horizon and more levels should be formed.

Thirdly, through the comprehensive evaluation system of enterprise “Internet +” cross-border connectivity, explore and study enterprise resources, capabilities, industry characteristics, and international experience and establish a scientific, objective, and systematic evaluation system.

## Figures and Tables

**Figure 1:** Market operation flow.

**Figure 2:** Mechanisms of experience in the Internet logistics industry.

**Figure 3:** Regional development trends in different.

**Figure 4:** Trade growth rates by year.

**Figure 5:** Overall growth rate of Belt and Road and growth rate over the previous year.

**Figure 6:** Distribution of growth rates by region versus total.

**Figure 7:** Growth rate fluctuation results and normalized error distribution after sample training.

**Figure 8:** Growth rate model prognosis evaluation analysis.

**Figure 9:** Growth rate of development power by country.

**Figure 10:** Share of countries in Internet logistics.

**Table 1:** Construction of the indicator system.

Tier-1 indicators	Tier-2 indicators	Tier-3 indicators
A: Information flow connection power	A_1_: Internet carriers	A_a1_: Internet penetration rate
		A_a2_: Fixed broadband subscriptions
		A_a3_: Mobile phone usage
		A_a4_: Number of secure Internet servers
	A_2_: Technical support	A_a5_: Exports of high technology products
		A_a6_: Technical readiness
		A_a7_: Innovation capacity

## Data Availability

The data used to support the findings of this study are available from the corresponding author upon request.
